The article "miR-26a and its Target CKS2 Modulate Cell Growth and Tumorigenesis of Papillary Thyroid Carcinoma" was retracted in 2021. Reasons: duplicated images; unreliable results or conclusions; concerns about the data; concerns about the images.

# miR-26a and its Target CKS2 Modulate Cell Growth and Tumorigenesis of Papillary Thyroid Carcinoma

**DOI:** 10.1371/journal.pone.0067591

**Published:** 2013-07-05

**Authors:** Mingli Lv, Xiaoping Zhang, Maoquan Li, Quanchi Chen, Meng Ye, Wenqing Liang, Lanbao Ding, Haidong Cai, Da Fu, Zhongwei Lv

**Affiliations:** 1 Department of Nuclear Medicine, Shanghai 10^th^ People’s Hospital, School of Medicine, Tongji University, Shanghai, China; 2 Department of Interventional Therapy, Shanghai 10^th^ People’s Hospital, School of Medicine, Tongji University, Shanghai, China; 3 Department of Orthopaedics, Shaoxing People’s Hospital, Shaoxing, China; H.Lee Moffitt Cancer Center & Research Institute, United States of America

## Abstract

**Background:**

While many studies have shown that levels of miR-26a are lower in papillary thyroid carcinoma (PTC), the role and mechanism of miR-26a in PTC are unclear.

**Method:**

We used database searches to select potential mRNA targets of miR-26a. Anti-miR-26a, miR-26a mimic, siRNA for CKS2 and their effects on cell growth, cell-cycle distribution and colony formation were evaluated. We also evaluate the over-expressed miR-26a in TPC-1 cells in severe combined immune-deficient mice. We used luciferase reporter assays, real-time PCR and western blot analysis to measure the expression and activity of miR-26a, CKS2, and related factors such as cyclin B1, cyclin A, cdk1, bcl-xl and Akt. Finally, we measured the relationship between the levels of miR-26a and CKS2 in PTC and normal thyroid tissues.

**Results:**

Relative to normal thyroid tissues, miR-26a is consistently down-regulated in TPC specimens, and CKS2 was identified as a potential target. Up-regulated miR-26a expression or down-regulated CKS2 expression in TPC-1 and CGTH W3 cells lines caused G2 phase-arrest. Decreased miR-26a expression or increased CKS2 expression could have inverse function on PTC cell lines. CyclinB1, cyclinA, bcl-xl and AKt are indirectly regulated by miR-26a in a CKS2-dependent manner. Finally, CKS2 is overexpressed in PTC specimens relative to normal thyroid tissue, and a significant inverse correlation exists between miR-26a and CKS2 expression in clinical PTC specimens.

**Conclusion:**

Our data indicate that miR-26a functions as a growth-suppressive miRNA in PTC, and that its suppressive effects are mediated mainly by repressing CKS2 expression.

## Introduction

Papillary thyroid carcinoma (PTC), which represents 70–80% of thyroid malignancies, generally has an excellent prognosis, even with cervical lymph node metastasis. Its prognosis is associated with age, tumor size, and histological parameters which include extracapsular extension, extrathyroidal extension, lymph node invasion distant metastasis and histological variants. These histological variants, which include conventional PTC, papillary thyroid microcarcinoma (PTMC), follicular variant (FVPC) and tall cell variant (TCVPC), among others, are related to familial adenomatous polyposis and tumor aggressiveness [1]. In addition, PTC is typically accompanied by gene rearrangement (e.g. *RET/PTC*) and/or sporadic mutation (e.g. *BRAF*) [2].

MicroRNAs (miRNAs) are ∼22 nucleotide length, non-coding single-stranded RNAs. To date, it has been estimated that miRNAs regulate the expression of about one-third of the mammalian protein-coding mRNAs, including mechanisms such as cleavage, resulting in 100% inhibition, as well as weaker forms of inhibition. Expression of miRNAs is subject to spatiotemporal regulation [3], and a number of miRNAs have been identified in various thyroid tumors, including PTC. Nikiforove et al. (4) used a ‘miRNACHIP’ micro-array approach to demonstrate that miR-187, −221, −222, −146b, −155, −122a, −31, −205 and −224 are up-regulated in PTCs compared with normal thyroid tissue. Chen et al. (5) also identified the upregulation of miR-146b, −221 and −222 in PTC. In total to date, 41 miRNAs have been shown to be over-expressed in thyroid carcinoma, including PTC, follicular thyroid carcinoma (FTC), medullary thyroid carcinoma (MTC) and anaplastic thyroid carcinoma (ATC) [4]. Conversely, a number of miRNAs which contribute to the development and progression of thyroid carcinoma are down-regulated in PTC, including miR-26a, −345,−138, −219, −218, −300, −292 and −30c [4], [5], [6], and in ATC, including miR-26a, −138, −219, −345, −30d and −125b [4], [7], [8].

As previously discussed, miRNA-microarray analysis has shown that miR-26a is down-regulated in PTC tissue relative to adjacent normal tissue by miRNA-microarray analysis [5]. miR-26a appears to have opposing functions in tumor growth in various types of cancer, acting as a tumor suppressor in renal cancer, lung cancer, breast cancer and liver cancer, but functioning as an oncogene in glioma [9], [10], [11], [12], [13]. Until now, the mechanism of miR-26a in PTC has been unclear.

In order to arrive at a better understanding of PTC pathogenesis, we investigated the function of miR-26a in PTC. We used Internet databases (http://mirecords.biolead.org/, www.targetscan.org/, www.ncRNA.org/) to select potential mRNA targets, followed by dual-luciferase assays to validate these interactions. We tested the effects of miR-26a on cell growth, cell cycle distribution, colony formation and examined its role in PTC tumorigenesis in a mouse model. Finally, we examined the expression levels of miR-26a and its target gene, CKS2, in PTC and normal thyroid tissue.

## Materials and Methods

### Clinical Specimens

The research was approved by the Ethics Committee of Shanghai Tenth People's Hospital. All participant of the article provide their written informed consent to participate in this study. All experiments on animal were performed according to the Animal Experimental Ethics Committee of Tongji University China and approved by the Ethics Committee of Shanghai Tenth People's Hospital.

PTC tissues and normal thyroid tissues were obtained from patients undergoing resection of PTC or thyroid nodules at Shanghai Tenth People’s Hospital (Tongji University, Shanghai, China). Both tumor and normal tissues were histologically confirmed. No local or systemic treatment had been conducted prior to the operation. All tissues were snap frozen in liquid nitrogen at the time of surgical removal.

### Cell Culture and miRNA Transfection

The human PTC cell lines TPC-1 and CGTH W3 provided by the Chinese Academy of Medical were cultured in RPMI-1640 containing 10% fetal bovine serum, 100 U/Ml penicillin and 100 µg/mL streptomycin. HEK-293T cells were grown in DMEM (Invitrogen) containing 10% fetal bovine serum from North American. Lipofectamine 2000 (Invitrogen) were used to transfect miRNAs and vectors according to the manufacturer’s instructions. The miR-26a mimic, a nonspecific miR control, anti-miR26a, a nonspecific anti-miR control, siRNA for CKS2 and a nonspecific siRNA control were all purchased from Sigma Company.

### Selected Targets mRNA for miR-26a

Target mRNAs for miR-26a were predicted using Targetscan (www.targetscan.org/), ncRNA (www.ncRNA.org/) and mirecords (http://mirecords.biolead.org/). In order to qualify as a target, the target mRNA had to contain at least one predicted miR-26a target site in its 3′UTR according to all three prediction algorithms. Gene Ontology (GO) was used in a subsequent screening step. We determined that the 3′-UTR of CKS2 was the best candidate target mRNA.

### Vector Construction and Luciferase Reporter Assays

Luciferase reporter assays were carried out using the Dual-Luciferase Reporter Assay System (psiCHECK-2 vector, Promega). A fragment of 3′UTR of CKS2 (278 bp) containing the putative miR-26a binding site was amplified by PCR using the following primers:

wt-CKS2 (forward) 5′ AAA-CTCGAG-AAGATTTGACATTCCCCA 3′

wt-CKS2 (reverse) 5′ CCC-GCGGCC-GTTCGACTTTACCTGTACT 3′

The PCR product was subcloned into the psiCHECK-2 vector downstream of the luciferase gene sequence. At the same time, a psiCHECK-2 vector containing 3′UTR of CKS2 with a mutant seed sequence of miR-26a was synthesized using the following primers:

Mut-CKS2 (forward) 5′ TCAGTGAATATCCGAGAAATG 3′

Mut-CKS2 (reverse) 5′ TTGTACATTTCTCGGCTATT 3′

A PLL3.7 vector (Invitrogen) containing the miR-26a sequence (200 bp) was also synthesized using the following primers, and named miR-26a- PLL3.7. Restriction enzyme sites were added at upstream (HpaI) and downstream (XhoI) positions.

miR-26a (forward) 5′ AA-GTTAAC-GTGGCCTCGTTCAAGTAATCCAGGATA GGCTGT 3′

miR-26a (reverse) 5′ AA-CTCGAG-AGCCTATCCTGGATTACTTGAACGAGG CCACG 3′

All constructs were verified by DNA sequencing. HEK-293 cells were plated in 96-well clusters, after which psiCHECK-2 vector containing wt- or mut-CKS2 was co-transfected with 100 ng construct with or without miR-26a precursors. Forty-eight hours after transfection, luciferase activity was detected using a dual-luciferase reporter assay system and normalized to Renilla activity.

In addition we also constructed the PMCB vector, which contains CKS2 (marked as CKS2-PMCB) using the following primers. The procedure was similar to that used for miR-26a-PLL3.7. Restriction enzyme sites were added at upstream (EcoRI) and downstream (BamHI) positions.

CKS2-PMCB (forward): AAA-GAATTC-ACGAGGATGGCCCACAAG

CKS2-PMCB (reversed): AAA-GGATCC-CATTTTTGTTGATCTTTTGG

### mRNA Expression Profiling

**RNA isolation:** Total RNA was isolated using Trizol reagent (Invitrogen) following the manufacturer’s instructions, and stored at −80°C. **Reverse transcription:** For miR-26a expression, total RNA was polyadenylated and reverse-transcribed using an NCode miRNA First-Strand cDNA Synthesis kit (Invitrogen). For CKS2 and β-Actin, total RNA was reversely transcribed using ImProm-II Reverse Transcription System (Promega). **Quantitative:** Real-time PCR analysis: qRT-PCR was performed following a standard SYBR-Green PCR kit protocol on a Step One Plus system (Applied Biosystems). β-Actin was used as an endogenous control to normalize the amount of total mRNA or miRNA in each sample, and relative expression was calculated with the comparative CT method.

### Western Blot Analysis

Equal amounts of cell lysates were separated by 10% SDS-PAGE, and electrophoretically transferred to PVDF membrane. The membrane was blocked and probed with mouse anti-human CKS2 monoclonal antibody (Abcam) followed by HRP (horseradish peroxidase)-labeled goat-antimouse IgG (Abcam). Chemiluminescence was used to analyze protein levels and β-Actin was used as a protein loading control.

### CCK-8 Cell Proliferation Assay

Cell proliferation rates were measured using a Cell Counting Kit (CCK-8) (Beyotime, Hangzhou, China). Twenty-four hours after cells were transfected with vectors, miR-26a mimic, anti-miR-26a, siRNA and their nonspecific controls, the cells were plated in 96-well plates at 500-cells per well. The cells were incubated for 24, 48, 72 or 96 h. Ten microliters of CCK-8 reagent was added to each well 1 h prior to detection. The OD 450 nm value in each well was determined by a microplate reader.

### Cell Cycle Analysis

The effects of miR-26a and its target gene on cell cycle progression were assessed using propidium iodide flow cytometry. Cells were plated in 6-well plates at 2×10^5^ per well and transfected with miRNAs, siRNA or vector. Seventy-two hours later, the cells were washed with PBS, harvested and fixed in 70% ethanol. Cells were treated with DNase-free RNase and stained with propidium iodide. Cell samples were analyzed on a FACSCalilur (BD Biosciences) and all cell cycle phase fractions were determined.

### Spheroid Formation Assay

Cells stably expressing miR-26a were transfected with anti-miR-26a, CKS2 siRNA or a nonspecific control. Twenty-four hours later, cells were seeded in 6-well plates at 200 per well. Two weeks later, colonies were washed twice using PBS, fixed with methanol/acetic acid, and stained in 1% crystal violet. The number of colonies was counted in four different field visions under a microscope and the mean value was taken.

### Apoptosis Flow Cytometry Analysis

Annexin V-FITC and propidium iodide flow cytometry using ApoAlert Annexin V kit (Clontech, Mountain View, CA) were used to assess the effects of miR-26a on cell death. TPC-1 cells and CGTH W3 cells stably expressing miR-26a, EV-control vector, with/without anti-miR-26a, siRNA for CKS2 and their nonspecific controls, were seeded in 6-well plates at 2×10^4^ per well. Cells were harvested 72 h later and stained with Annexin V-FITC and propidium iodide according to the manufacturer’s protocol. Cell samples were analyzed on a FACSCalibur and apoptotic fractions were determined.

### In vivo Tumorigenesis Assay

Male BALB/c nude mice (4 to 5 weeks of age) were purchased from the Animal Services Centre of Fudan University, China. All experiments on animal were performed according to the Animal Experimental Ethics Committee of Tongji University China. A total of 1×10^6 ^miR-26a-TPC-1 cells or PLL3.7-TPC-1 cells were injected into the dorsal flank of nude mice. Each group contained 6 mice and the experiment was repeated three times. Tumor size was measured every 2 days. The formula volume = (D×d^2^)/2 was used to evaluated tumor volume, where “D” is the longest diameter and “d” is the shortest diameter. Three weeks later, mice were sacrificed and the tumors dissected. The rate of growth of the tumor was analyzed by immunohistochemistry (ICH) for Ki-67 and PCNA, which is related to the increase in tumor size. The biopsy tissues were deparaffinized, dehydrated in xylene and graded alcohols, rinsed in PBS and stained by monoclonal antibodies for Ki-67 and PCNA (invitrogen Co.) at room temperature for 1 h, and then blocked by 3% H_2_O_2_ for 10 min at room temperature and washed thoroughly in PBS. Each tumor had at least three biopsy sections.

### Statistical Analysis

SPSS 15.0 software was used for statistical analysis. Data are expressed as the mean ± SEM, using a two-tail Student’s test to carry out comparisons of two independent groups. A *p*-value <0.05 was considered statistically significant. All experiments were performed in triplicate.

## Results

### Expression of miR-26a is Decreased in Clinical PTC Specimens

We compared miR-26a expression in 40 PTC specimens and 40 normal thyroid tissues. There were no significant differences in age, gender and the TNM tumor stage between two groups (Table 1). The average level of miR-26a was significantly lower in PTC specimens than in normal tissues (Fig. 1, *p* = 0.007).

**Figure 1:** Average expression levels of miR-26a and CKS2 in human PTC specimens (n = 40) vs. normal thyroid tissues (n = 40). **A.** miR-26a down-regulation in PTC specimens (n = 40) vs. normal thyroid tissues (n = 40) (*p*<0.001). **B.** Increased CKS2 expression increased in PTC specimens results shown by RT-PCR and western blot (*p* = 0.003).

**Table 1:** The clinical date of analyzed tissue samples.

		PTC	Normal	*p*
Average age		40.18±2.19	41.97±1.25	>0.05
Gender	F	19	18	>0.05
	M	21	22	

### mir-26a Inhibits Proliferation and Spheroid Formation, and Promotes Apoptosis, in TPC-1 and CGTH W3 Cells

To characterize the effect of miR-26a on cell proliferation we performed overexpression studies using a miR-26a mimic and inhibition studies using miR-26a specific anti-sense oligonucleotide inhibitor (anti-miR-26a). miR-26a inhibited, and anti-miR-26a promoted, cell proliferation in both TPC-1 cells and CGTH W3 cells (*p*<0.01)(Fig. 2A, Fig. S1). The nonspecific micro-RNA and anti-miR controls had no effect on cell growth in either cell line.

**Figure 2:** miR-26a inhibition of TPC-1 cell growth. **A.** Effect of miR-26a on TPC-1 cell proliferation measured by CCK8 assay. **B.** Effect of stable over-expression of miR-26a on TPC-1 cell proliferation measured by CCK8 assay. **C.** Expression of miR-26a in miR-26a-TPC-1 cells is higher than EV-TPC-1 cell and TPC-1 cell. **D.** Colony formation assay of TPC-1 cells transfected with miR-26a, miR control, anti-miR-26a, anti-miR control, and miR-26a-TPC-1 cell vs EV-TPC-1 cell. **E.** The relative numbers of colonies obtained by counting five vision fields. Error bars correspond to 95% confidence intervals. **F.** Cell-cycle distribution of TPC-1 cells transfected with miR-26a mimic, anti-mir-26a and their nonspecific controls for 48 h. **G.** Flow cytometry and Annexin V assays showing the number of cells in apoptosis in TPC-1 cells stably over-expressing miR-26a or control TPC-1 cells with blank PLL3.7 (EV-TPC-1 cell).

Next, we stably over-expressed miR-26a in TPC-1 (miR-26a-TPC-1) and CGTH W3 (miR-26a-CGTH W3) cells to examine its effect on cell growth. We first verified that expression levels of miR-26a were higher in miR-26a-TPC-1 cell and miR-26a-CGTH W3 cell than in control or untreated cells (Fig. 2C, Fig. S2). The growth inhibition effected by lentivirally-expressed miR-26a was similar to that induced by miR-26a mimic transfection in both cell lines (*p*<0.001, Fig. 2B, Fig. S3). Collectively these studies indicated that miR-26a modulates PTC cell growth. Next we showed that miR-26a over-expression decreases colony formation efficiency in TPC-1 cells (Figs. 2D and E), and that anti-miR-26a increased colony formation capacity in TPC-1 cell lines (Figs. 2D and E). The control lentivirus vector had no effect on cell colony formation. This result demonstrates that miR-26a modulates PTC cell colony formation capacity.

In order to explore the mechanism of miR-26a in cellular proliferation, we examined its effect on cell cycle distribution and apoptosis. First we transfected TPC-1 and CGTH W3 cells with a miR-26a mimic, or anti-miR-26a, and examined their effects on cell cycle distribution. Overexpression of miR-26a significantly increased the number of cells in G_2_ phase in both cell lines (*p*<0.01, Fig. 2F, Fig. S4) compared with its nonspecific miRNA control. The number of anti-miR-26a-transfected cells in the G_2_ phase was significantly decreased compared with the nonspecific anti-miRNA-transfected controls in both cell lines. Flow cytometry and Annexin V assay results demonstrated that apoptosis was significantly increased in miR-26a stably-overexpressed TPC-1 and CGTH W3 cells compared to cells transfected with empty PLL3.7 (*p*<0.01, Fig. 2G, Fig. S5). These data indicate that the growth-suppressive effect of miR-26a is due to G_2_ phase-arrest and increased apoptosis.

### CKS2 is a Target of miR-26a

To explore mi-26a-regulated target gene(s) and pathway(s), we used three publicly-available miRNA target prediction tools: Targetscan, ncRNA and mirecords. To increase the stringency of the target prediction protocol, we searched for mRNAs simultaneously predicted by all the three target-prediction programs and selected CKS2 as a potential target. To assess whether miR-26a could directly alter the expression of CKS2, a fragment of the 3′UTR of CKS2 mRNA (wt 3′UTR) containing the putative miR-26a binding sequence (or the mutant sequence, mut 3′UTR), was cloned into a luciferase reporter vector (Fig. 3A). HEK-293T cells were then transfected with the wild type or mut 3′UTR of CKS2 and miR-26a mimic. As shown in Fig. 3A, luciferase expression was decreased by about 50% when the wt 3′UTR and miR-26a mimic were cotransfected, while the mut 3′UTR had no effect on luciferase activity. Moreover cotransfection of HEK-293T cells with the wt 3′UTR and anti-miR-26a reversed the decrease caused by the miR-26a mimic (Fig. 3B). Collectively, these results indicate that CKS2 is a direct target of miR-26a.

**Figure 3:** CKS2 is a target of miR-26a and miR-26a regulates CKS2 downstream signaling molecules. **A.** Putative binding site of miR-26a on the CKS2 3′UTR along with the mutation in the predicted seed region. **B.** Reporter assays on HEK-293T cells transfected with the reporter vectors containing either the wildtype or mutated CKS2 3′UTR. **C.** Protein levels of CKS2 in TPC-1 cells transfected with miR-26a mimic, anti-miR-26a or their nonspecific controls. **D.** miR-26a mediated reduction of CKS2 levels is associated with decreased expression of cyclinB1 and cdk1, and increased expression of bcl-xl and Akt, shown by RT-PCR and western blot. **E.** siRNA for CKS2 decreases expression of cyclinB1 and cdk1, and increases expression of bcl-xl and Akt, shown by RT-PCR and western blot. **F.** Transfection with anti-miR-26a increases cyclin B1 and cdk1 expression, and decreases bcl-xl and Akt expression, as shown by RT-PCR and western blot.

Since microRNAs regulate cell function in a spatiotemporal fashion, we next elucidated whether the growth-suppressive effect of miR-26a was mediated by repression of CKS2 in TPC-1 and CGTH W3 cells. We first verified whether expression of CKS2 changed in response to transfection with miR-26a mimic or anti-miR-26a. Compared to controls, expression of CKS2 was significantly decreased by miR-26a transfection and increased by anti-miR-26a transfection (Fig. 3C), indicating that miR-26a decreases CKS2 expression in TPC-1 cells.

### CKS2 siRNA Inhibits Proliferation and Spheroid Formation, and Promotes Apoptosis, in TPC-1 and CGTH W3 Cells

Next we silenced CKS2 expression in TPC-1 and CGTH W3 cells to determine whether the effect of reduced expression of CKS2 was similar to that of miR-26a. TPC-1 cells and CGTH W3 cells were transfected with siRNA for CKS2 or a miR-26a mimic. In the CCK8 cell proliferation assay, CKS2 knockdown led to significant cell growth inhibition, similar to that induced by miR-26a transfection (Fig. 4A). Moreover, cell colony formation efficiency decreased after transfection with CKS2 siRNA to an extent comparable to that induced by miR-26a (Fig. 4B). Furthermore, knockdown of CKS2 resulted in a increase in the number of cells in the G_2_ phase and, like transfection with miR-26a, promoted TPC-1 cell apoptosis (Figs. 4C and D, Fig. S6 and S7).

**Figure 4:** Knockdown of CKS2 inhibits TPC-1 cell growth. **A.** Effect of miR-26a transfection or CKS2 knockdown on TPC-1 cell proliferation measured by CCK8 assay. **B.** Colony formation assay of TPC-1 cells transfected with miR-26a mimic, miR control, CKS2 siRNA and siRNA control, and the relative numbers of colonies counted under a microscope in five vision fields. Error bars correspond to 95% confidence intervals. **C.** Cell-cycle distribution of TPC-1 cells transfected with miR-26a mimic, miR control, CKS2 siRNA and siRNA control for 48 h. **D.** Flow cytometry and annexin V assays reflect the number of apoptotic TPC-1 cells after transfection with miR-26a mimic, miR control, CKS2 siRNA or siRNA control.

Next we determined whether up-regulation of CKS2 had a similar effect to that of anti-miR-26a. Similar to the effects of anti-miR-26a, CKS2 overexpression increased cell proliferation and colony formation efficiency, and decreased the number of cells in G_2_ phase and apoptosis (Fig. 5). In summary, these results indicate that CKS2 is a downstream target gene of miR-26a, and that the growth-suppressive effect of miR-26a is mediated by repression of CKS2 in TPC-1 cells.

**Figure 5:** Stable over-expressison of CKS2 and anti-miR-26a promotes TPC-1 cell growth. **A.** Effects of CKS2 or anti-miR-26a over-expression on TPC-1 cell proliferation. CKS2 = TPC-1 cell transfected with CKS2-PMCB vector; EV = TPC-1 cell transfected with EV-PMCB vector. **B.** Colony formation assay of TPC-1 cells transfected with CKS2-PMCB, EV-PMCB, anti-miR-26a and anti-miR control, and the relative numbers of colonies counted under microscope in five vision fields. Error bars correspond to 95% confidence intervals. **C.** Cell-cycle distribution of TPC-1 cells transfected with CKS2-PMCB, EV-PMCB, anti-miR-26a and anti-miR control for 48 h. **D.** Flow cytometry and Annexin V assays reflect the number of apoptotic TPC-1 cells after transfection with CKS2-PMCB, EV-PMCB, anti-miR-26a and anti-miR control.

### CKS2 Overexpression Rescues the Growth Suppressive Effect of miR-26a

In order to prove that miR-26a exerts its growth inhibitory effects by inhibiting CKS2 expression, we also performed the rescued experiment. In the experiment, miR-26a-TPC-1 cells which stably over-expressing miR-26a were transient transfected with CKS2-PMCB or EV-PMCB. The cells transfected with CKS2-PMCB had stronger ability of proliferation and monoclonal formation (Fig. 6A and Fig. 6B). Furthermore transfected with CKS2-PMCB resulted in a decrease in the number of cells in the G2 phase and inhibited both cells apoptosis (Fig. 6C and Fig. 6D). All these results indicated that CKS2 overexpression could rescue the growth suppressive effect of miR-26a. MiR-26a exerts its growth inhibitory effects and promoted apoptosis by inhibiting CKS2 expression.

**Figure 6:** CKS2 overexpression rescues the growth suppressive effect of miR-26a. **A.** Effects of CKS2 over-expression on miR-26a-TPC-1 cell proliferation. MiR-26a+CKS2 = miR-26a-TPC-1 cell transfected with CKS2-PMCB vector; MiR-26a +EV = miR-26a-TPC-1 cell transfected with EV-PMCB vector. **B.** Colony formation assay of miR-26a-TPC-1 cells transfected with CKS2-PMCB or EV-PMCB, and the relative numbers of colonies counted under microscope in five vision fields. Error bars correspond to 95% confidence intervals. **C.** Cell-cycle distribution of miR-26a-TPC-1 cells transfected with CKS2-PMCB or EV-PMCB for 48 h. **D.** Flow cytometry and Annexin V assays reflect the number of apoptotic miR-26a-TPC-1 cells after transfection with CKS2-PMCB, or EV-PMCB.

### miR-26a Suppresses Tumor Growth of TPC-1 Cells in vivo

TPC-1 cells stably infected with miR-26a or a control vector were injected into the dorsal flank of nude mice. About 1 week after inoculation, the tumors became palpable. All mice had developed tumors by the end of 3 weeks. Eleven days after implantation, the average volume of transplanted tumors between the two groups became statistically significant, and miR-26a-PLL3.7 infected cells produced smaller tumors than control cells (Fig. 7A). At 17 days post-implantation, the average tumor volume of the miR-26a-PLL3.7 treated group was reduced by more than 50% compared with those treated with control TPC-1 cells (Fig. 7A). When mice were sacrificed 3 weeks post-implantation, the average weight of tumors in the miR-26a treated group was significantly less than the control (Fig. 7B). IHC analysis showed that miR-26a-treated mice had lower levels of Ki-67 and PNCA than control mice, indicating a lower tumor growth rate in miR-26a-transfected tumor cells (Fig. 7C). In summary, miR-26a suppressed the tumor growth of TPC-1 cell in nude mice.

**Figure 7:** miR-26a suppresses tumor growth of TPC-1 cells in nude mice. **A.** Growth curve of tumors volumes over 21 days of observation. Each data point represents the mean ± SEM of six mice. **B.** The tumors were dissected from the mice and measured. **C.** IHC Ki-67 and PNCA staining of sections of transplanted tumors formed by TPC-1 cells infected with miR-26a-PLL3.7 or EV-PLL3.7.

### miR-26a Regulates CKS2 Downstream Signaling Molecules

Given that miR-26a suppressed tumor cell proliferation and promoted apoptosis through inhibition of CKS2 expression, we examined the effect of miR-26a on CKS2 downstream signaling molecules in our system. Cyclin B1, Cyclin A, cdk1, bcl-xl and AKt were selected as CKS2 downstream genes [14], [15]. miR-26a-mediated reduction of CKS2 levels was associated with decreased expression of cyclinB1, cdk1, bcl-xl and AKt expression (Fig. 3D). Similarly, these genes expression was increased,in CKS2 siRNA-transfected TPC-1 cells (Fig. 3E). Conversely, transfection of anti-miR-26a resulted in elevated expression levels of cyclinB1, cdk1, bcl-xl and AKt (Fig. 3F). These results implicate cyclin B1, cdk1, bcl-xl and AKt in miR-26a-mediated tumor growth suppression.

### CKS2 Expression is Increased in Clinical PTC Specimens and is Inversely Correlated with miR-26a Levels

In order to evaluate the clinical implications of the relationship between miR-26a and CKS2 we identified in our *in vitro* experiments, we next measured the expression levels of CKS2 in PTC specimens and normal thyroid tissues. As showed in Fig. 1B, average expression levels of CKS2 were significantly higher in PTC specimens than in normal thyroid tissues (*p*<0.05). Moreover, as anticipated, we observed a significant inverse correlation between CSK2 and miR-26a levels (Fig. 1C, r = −0.964; *p*<0.001) in these tissues.

## Discussion

PTC is the most common form of follicular-cell derived carcinomas and comprises 75% of all newly-diagnosed thyroid cancers [16]. While studies have shown that miR-26a is down-regulated in PTC [4], [5], [6], [7], [8], to date no data have been available regarding the mechanism of miR-26a in this disease. miR-26a has been shown to inhibit tumor cell growth in an EZH2-dependent manner in nasopharyngeal carcinoma [17], and a similar pathway has been demonstrated in lung cancer [10]. Moreover, mir-26a promotes cholangiocarcinoma growth through activation of β-catenin [13]. It is known however that a given miRNA may target several mRNAs, and that miRNAs have tissue specific functions, and these functions may not be conserved across different tumor types.

In this study we first validated that miR-26a was down-regulated in PTC specimens compared to normal thyroid tissues. We then tested the effects on various parameters of cell growth of miR-26a transfection in our TPC-1 and CGTH W3 cell line PTC models, and found that miR-26a overexpression inhibited TPC-cell proliferation, decreased clonogenic formation, induced G_2_-arrest and promoted apoptosis. Conversely, in the same cell models, anti-miR-26a promoted cell proliferation and clonogenic formation, and inhibited apoptosis. IHC analysis of Ki-67 and PCNA demonstrated that overexpression of miR-26a suppressed tumorigenesis in a murine model of TPC-1 xenograft, echoing similar findings in nasopharyngeal carcinoma, lung cancer, liver cancer [18] and lymphoma [19]. In all these studies, miR-26a was down-regulated, and re-established expression of miR-26a inhibited cell proliferation and promoted apoptosis. In cholangiocarcinoma and glioma however, miR-26a acts as an oncogene to promote cell growth [11], [13]. These conflicting data indicate that the expression and action of miR-26a is tissue- and time- dependent, and its role in different tumor cells may potentially alter according to its downstream targets.

Cyclin-dependent kinase subunit (Cks) proteins are small cyclin-dependent kinase-interacting proteins which are essential for cell cycle control [20], [21]. The mammalian Cks family consists of two well-conserved small proteins, Cks1 and Cks2 (also referred to as CDC28 protein kinase regulatory subuinit2, or CKS2). Many human malignancies are characterized by CKS2 overexpression, and it is generally known as an oncogene. In our study, a variety of results indicated that CKS2 is a direct target of miR-26a in TPC-1 cells: (i) a seed binding site sequence for miR-26a was identified in the 3′UTR of CKS2 mRNA; (ii) CKS2 3′UTR luciferase reporter activity was decreased by overexpression of miR-26a but not by mut-miR-26a, contains a mutation in the seed binding site of miR-26a; (iii) CKS2 mRNA and protein levels were decreased by miR26a overexpression in TPC-1 and CGTH W3 cells, and this effect was attenuated by anti-miR-26a; (iv) silencing CKS2 expression in TPC-1 cells had similar cell-growth suppressive effects to those of overexpression of miR-26a; (v) CKS2 overexpression rescued the growth suppressive effect of miR-26a to an extent similar to that of anti-miR-26a; and (vi) a significant inverse correlation exists between miR-26a and CKS2 in clinical PTC specimens. Collectively, these results suggest that the growth inhibitory effect of miR-26a is mediated via repression of CKS2 expression.

In order to further explore the molecular mechanism of the growth inhibition induced by miR-26a, we examined its effect on the expression of a panel of CKS2 downstream genes, namely cyclinB1, cyclin A, cdk1, bcl-xl and Akt [14], [15]. Our results showed that cyclinB1, cyclin A, bcl-xl and AKt were regulated by miR-26a and CKS2. Cdk1 and cyclin B1 are known to be important players in the cell cycle. Many studies have demonstrated that Cyclin B1-cdk1 protein kinase, also known as mitosis promoting factor (MPF), is essential for mitosis and that in its absence, cells are unable to progress past the G2 phase of the cell cycle [22], [23]. Consistent with this, we found that the growth-suppressive effect of miR-26a was partly due to a G_2_ phase-arrest. Together, these data are consistent with a model in which miR-26a suppresses CKS2 expression, leading to suppressed of cyclin B1 and cdk1 expression and G_2_ arrested, similar to the findings of a previous study [15]. Moreover, consistent with the previous data [16], our results indicate that miR-26a induced cell apoptosis involves by Bcl-xl and Akt, which are mainly involved in programmed cell death.

In summary, this study provides novel evidence that in a model of papillary thyroid carcinoma, miR-26a suppresses proliferation and colony formation efficiency, induces G_2_ cell cycle arrest, promotes cell apoptosis and inhibits tumor growth in vivo by targeting CKS2 and ultimately regulating the expression of cyclinB1, cdk1, bcl-xl and AKt. Moreover, there is a significant inverse correlation between miR-26a and CKS2 in clinical PTC specimens. Our findings suggest that signaling molecules in this pathway might represent potential targets for future prevention and treatment of human papillary thyroid carcinoma.

## Supporting Information

Figure S1 **Effect of miR-26a on CGTH W3 TPC-1 cell proliferation measured by CCK8 assay.**
(TIF)

Figure S2 **Expression of miR-26a in miR-26a-transfected CGTH W3 cells is higher than in EV- CGTH W3 cell and CGTH W3 cell.**
(TIF)

Figure S3 **The effect of stable over-expression of miR-26a on CGTH W3 cells proliferation measured by CCK8 assay.**
(TIF)

Figure S4 **Cell-cycle distribution of CGTH W3 cells transfected with miR-26a mimic, anti-mir-26a and their nonspecific control for 48 h.**
(TIF)

Figure S5 **Flow cytometry and Annexin V assays show the number of apoptotic CGTH W3 cells after stable over-expression of miR-26a (miR-26a-CGTH W3 cell) compared to mock-transfected CGTH W3 cells (PLL3.7- CGTH W3 cell).**
(TIF)

Figure S6 **Cell-cycle distribution of CGTH W3 cells transfected with miR-26a mimic, miR control, CKS2 siRNA or siRNA control for 48 h.**
(TIF)

Figure S7 **Flow cytometry and Annexin V assays show the number of apoptotic TPC-1 cells transfected with miR-26a mimic, miR control, CKS2 siRNA or siRNA control.**
(TIF)

## References

[1] Gonzalez-GonzalezR, Bologna-MolinaR, Carreon-BurciagaRG, Gomezpalacio-GastelumM, Molina-FrecheroN, et al (2011) Papillary thyroid carcinoma: differential diagnosis and prognostic values of its different variants: review of the literature. ISRN Oncol 2011: 915925.2243205410.5402/2011/915925PMC3302055

[2] BartelDP, ChenCZ (2004) Micromanagers of gene expression: the potentially widespread influence of metazoan microRNAs. Nat Rev Genet 5: 396–400.1514332110.1038/nrg1328

[3] SchmittgenTD, LivakKJ (2008) Analyzing real-time PCR data by the comparative C(T) method. Nat Protoc 3: 1101–1108.1854660110.1038/nprot.2008.73

[4] PallanteP, VisoneR, CroceCM, FuscoA (2010) Deregulation of microRNA expression in follicular-cell-derived human thyroid carcinomas. Endocr Relat Cancer 17: F91–104.1994271510.1677/ERC-09-0217

[5] HeH, JazdzewskiK, LiW, LiyanarachchiS, NagyR, et al (2005) The role of microRNA genes in papillary thyroid carcinoma. Proc Natl Acad Sci U S A 102: 19075–19080.1636529110.1073/pnas.0509603102PMC1323209

[6] TetzlaffMT, LiuA, XuX, MasterSR, BaldwinDA, et al (2007) Differential expression of miRNAs in papillary thyroid carcinoma compared to multinodular goiter using formalin fixed paraffin embedded tissues. Endocr Pathol 18: 163–173.1805826510.1007/s12022-007-0023-7

[7] MitomoS, MaesawaC, OgasawaraS, IwayaT, ShibazakiM, et al (2008) Downregulation of miR-138 is associated with overexpression of human telomerase reverse transcriptase protein in human anaplastic thyroid carcinoma cell lines. Cancer Sci 99: 280–286.1820126910.1111/j.1349-7006.2007.00666.xPMC11159409

[8] VisoneR, PallanteP, VecchioneA, CirombellaR, FerracinM, et al (2007) Specific microRNAs are downregulated in human thyroid anaplastic carcinomas. Oncogene 26: 7590–7595.1756374910.1038/sj.onc.1210564

[9] ChenHC, ChenGH, ChenYH, LiaoWL, LiuCY, et al (2009) MicroRNA deregulation and pathway alterations in nasopharyngeal carcinoma. Br J Cancer 100: 1002–1011.1929381210.1038/sj.bjc.6604948PMC2661776

[10] DangX, MaA, YangL, HuH, ZhuB, et al (2012) MicroRNA-26a regulates tumorigenic properties of EZH2 in human lung carcinoma cells. Cancer Genet 205: 113–123.2246951010.1016/j.cancergen.2012.01.002

[11] HuseJT, BrennanC, HambardzumyanD, WeeB, PenaJ, et al (2009) The PTEN-regulating microRNA miR-26a is amplified in high-grade glioma and facilitates gliomagenesis in vivo. Genes Dev 23: 1327–1337.1948757310.1101/gad.1777409PMC2701585

[12] Slaby O, Redova M, Poprach A, Nekvindova J, Iliev R, et al. Identification of MicroRNAs associated with early relapse after nephrectomy in renal cell carcinoma patients. Genes Chromosomes Cancer 51: 707–716.2249254510.1002/gcc.21957

[13] Zhang J, Han C, Wu T (2012) MicroRNA-26a promotes cholangiocarcinoma growth by activating beta-catenin. Gastroenterology 143: 246–256 e248.10.1053/j.gastro.2012.03.045PMC366833622484120

[14] LanY, ZhangY, WangJ, LinC, IttmannMM, et al (2008) Aberrant expression of Cks1 and Cks2 contributes to prostate tumorigenesis by promoting proliferation and inhibiting programmed cell death. Int J Cancer 123: 543–551.1849813110.1002/ijc.23548PMC3262990

[15] Martinsson-AhlzenHS, LiberalV, GrunenfelderB, ChavesSR, SpruckCH, et al (2008) Cyclin-dependent kinase-associated proteins Cks1 and Cks2 are essential during early embryogenesis and for cell cycle progression in somatic cells. Mol Cell Biol 28: 5698–5709.1862572010.1128/MCB.01833-07PMC2546922

[16] BanY, YamamotoG, TakadaM, HayashiS, ShimizuK, et al (2012) Proteomic profiling of thyroid papillary carcinoma. J Thyroid Res 2012: 815079.2251834810.1155/2012/815079PMC3306988

[17] LuJ, HeML, WangL, ChenY, LiuX, et al (2011) MiR-26a inhibits cell growth and tumorigenesis of nasopharyngeal carcinoma through repression of EZH2. Cancer Res 71: 225–233.2119980410.1158/0008-5472.CAN-10-1850

[18] JiJ, ShiJ, BudhuA, YuZ, ForguesM, et al (2009) MicroRNA expression, survival, and response to interferon in liver cancer. N Engl J Med 361: 1437–1447.1981240010.1056/NEJMoa0901282PMC2786938

[19] SanderS, BullingerL, KlapprothK, FiedlerK, KestlerHA, et al (2008) MYC stimulates EZH2 expression by repression of its negative regulator miR-26a. Blood 112: 4202–4212.1871394610.1182/blood-2008-03-147645

[20] HaylesJ, BeachD, DurkaczB, NurseP (1986) The fission yeast cell cycle control gene cdc2: isolation of a sequence suc1 that suppresses cdc2 mutant function. Mol Gen Genet 202: 291–293.301005110.1007/BF00331653

[21] RichardsonHE, StuelandCS, ThomasJ, RussellP, ReedSI (1990) Human cDNAs encoding homologs of the small p34Cdc28/Cdc2-associated protein of Saccharomyces cerevisiae and Schizosaccharomyces pombe. Genes Dev 4: 1332–1344.222741110.1101/gad.4.8.1332

[22] DoreeM, HuntT (2002) From Cdc2 to Cdk1: when did the cell cycle kinase join its cyclin partner? J Cell Sci 115: 2461–2464.1204521610.1242/jcs.115.12.2461

[23] VassilevLT, TovarC, ChenS, KnezevicD, ZhaoX, et al (2006) Selective small-molecule inhibitor reveals critical mitotic functions of human CDK1. Proc Natl Acad Sci U S A 103: 10660–10665.1681888710.1073/pnas.0600447103PMC1502288

